# Diagnostic Value of Coronary Computed Tomography Angiography Image under Automatic Segmentation Algorithm for Restenosis after Coronary Stenting

**DOI:** 10.1155/2022/7013703

**Published:** 2022-04-16

**Authors:** Xinrong He, Juan Zhao, Yunpeng Xu, Huini Lei, Xianbin Zhang, Ting Xiao

**Affiliations:** ^1^Department of Cardiovascular Medicine 7, Xianyang Hospital of Yan'an University, Xianyang 712000, Shaanxi, China; ^2^Department of Cardiovascular Medicine 2, Xianyang Hospital of Yan'an University, Xianyang 712000, Shaanxi, China; ^3^Interventional Operating Room, Shangluo Central Hospital, Shangluo 726000, Shaanxi, China; ^4^Department of Cardiology, Xi'an Changan Hospital, Xi'an 710000, Shaanxi, China; ^5^Department of Cardiovascular Medicine, Shangluo Central Hospital, Shangluo 726000, Shaanxi, China

## Abstract

The diagnostic efficacy of coronary computed tomography angiography (CTA) images of coronary arteries in restenosis after coronary stenting based on the combination of the convolutional neural network (CNN) algorithm and the automatic segmentation algorithm for region growth of vascular similarity features was explored to provide a more effective diagnostic method for patients. 130 patients with coronary artery disease were randomly selected as the research objects, and they were averagely classified into the control group (conventional coronary CTA image diagnosis) and the observation group (coronary CTA image diagnosis based on an improved automatic segmentation algorithm). Based on the diagnostic criteria of coronary angiography (CAG), the efficacy of two kinds of coronary CTA images on the postoperative subsequent visit of coronary heart disease (CHD) stenting was evaluated. The results showed that the accuracy of the CNN algorithm was 87.89%, and the average voxel error of the improved algorithm was signally lower than that of the traditional algorithm (1.8921 HU/voxel vs. 7.10091 HU/voxel) (*p* < 0.05). The average score of the coronary CTA image in the observation group was higher than that in the control group (2.89 ± 0.11 points vs. 2.01 ± 0.73 points) (*p* < 0.05). The diagnostic sensitivity (91.43%), specificity (86.76%), positive predictive value (88.89%), negative predictive value (89.66%), and accuracy (89.23%) of the observation group were higher than those of the control group (*p* < 0.05). In conclusion, the region growth algorithm under the CNN algorithm and vascular similarity features had an accurate segmentation effect, which was helpful for the diagnosis of CTA image in restenosis after coronary stenting.

## 1. Introduction

With the rapid development of science and technology, economy, and culture, the types of diseases also increase. Due to the changes in people's daily living habits, the incidence of many diseases is increasing, and coronary heart disease (CHD) is one of them. In recent years, the incidence of CHD has increased with the trend of patients being young and the aging of the population [1, 2]. Angina pectoris and other symptoms of CHD bring great pain to patients [3, 4]. Coronary stent implantation is one of the most effective therapies at present [5]. About 2 million patients with CHD worldwide are treated with coronary stent implantation every year [6]. However, in-stent restenosis (ISR) occurs in some patients after surgery. Hence, rediagnosis is more crucial for these patients. The “gold standard” for the diagnosis of ISR is coronary angiography (CAG) [7]. Nevertheless, this method is not well accepted by patients because it is expensive, invasive, and the operation is complex. Nonetheless, coronary computed tomography angiography (CTA) [8] is a preferred method for people with simple operations, noninvasive examinations, and low inspection costs [9]. Besides, coronary CTA has a good diagnosis effect on CHD and postoperative restenosis [10].

In the past, CTA images of patients in clinical practice were examined or reviewed by doctors who observed the lesions through artificial segmentation [11]. Nevertheless, this method often causes the interference of subjective consciousness in the examination results, which leads to errors in the diagnosis results of diseases that can reduce the diagnostic accuracy [12]. To solve the abovementioned problems, an automatic segmentation technology is proposed through continuous exploration [13]. After continuous adoption and research, automatic segmentation technology has become a vital auxiliary means in the diagnosis of coronary CTA images for CHD. The segmentation algorithm is mainly classified into image denoising and image segmentation [14]. The segmentation algorithm based on the growth algorithm [15] is relatively ubiquitous. This method uses the similarity of pixels in different regions to classify regions, but the accuracy of segmentation is low [16]. Therefore, this method needs to be improved.

To sum up, coronary CTA images based on an improved automatic segmentation algorithm were employed for postoperative coronary stenting reexamination. The diagnostic value of CAG was evaluated with the diagnostic results as the gold standard to provide more accurate and effective examination methods for patients with CHD so that they could receive reasonable treatment.

## 2. Materials and Methods

### 2.1. Objects of Study

In this study, 130 patients who came to the hospital for the postoperative subsequent visit of CHD stenting between March 2019 and March 2021 were randomly selected as the research objects. There were 90 male patients and 40 female patients. The patients were 30–80 years old and the average age was 60.21 ± 9.55 years old. The diameter of the stent was 2mm–4 mm with an average diameter of 2.86 ± 0.19 mm. By the random number table, all the patients were classified into the control group (conventional coronary CTA image diagnosis) and the observation group (coronary CTA image diagnosis based on the improved automatic segmentation algorithm), each of which included 65 cases. The diagnostic results of CAG were taken as the standard to evaluate the effect of two kinds of CTA images on the postoperative subsequent visit of CHD stenting. This study has been approved by the ethics committee of the hospital. Patients and their families were aware of this research and signed informed consent.

The inclusion criteria were as follows: (i) patients who agreed to the CAG examination; (ii) patients whose reexamination was within 3 months after surgery; (iii) patients who signed the informed consent; and (iv) patients with single-vessel lesion.

The exclusion criteria were as follows: (i) patients with severe heart, liver, and renal insufficiency; (ii) patients who were allergic to iodine-containing contrast agents; (iii) patients with contraindications to coronary CTA examination; (iv) patients with hyperthyroidism; and (v) patients whose conditions were unstable.

### 2.2. Methods of Examination

#### 2.2.1. The CAG Examination

Coronary angiography was performed by a digital subtraction angiography system for CAG. After the F sheath tube was introduced through radial artery puncture, 3,000–5,000 u of heparin as the anticoagulant was injected through the sheath tube before the imaging surgery. After the heparin injection was completed, an iodine-containing contrast agent (Ultravist) was injected by a Radial 5F TIG angiography catheter to perform angiography for the left and right coronary arteries. There were 6 positions of left coronary angiography, which were positive: left anterior oblique, right anterior oblique, spider, liver, and foot. Right coronary angiography was performed in two positions. One was the left anterior oblique position, and the other was head posture. The collected images were evaluated by several senior coronary interventional physicians. The evaluation methods were mostly visual observation.  Figure 1 shows the evaluation criteria for ISR.

#### 2.2.2. Coronary CTA Examination

Coronary CTA was examined by a 64-slice spiral CT. During the examination, the patient was placed in the supine position, and electrocardiogram (ECG) monitoring was required. The scanning range was from 1.4 cm below the tracheal bifurcation to 2 cm below the diaphragmatic surface of the heart. A contrast agent (pump speed: 5 mL/s and contrast agent: iohexol) was injected with a high-pressure syringe, and the dose was controlled at 55–70 mL according to the patient's weight. The injection time was 11 s–14 s. After that, 35 mL of normal saline was injected. Then, automatic scanning was performed, and images of each vessel were collected. Specific scanning parameters were as follows: tube voltage was −120 kV; tube current was −320 mA; revolving speed was −0.37 s/r; layer thickness was −0.65 mm; and pitch was −0.19. The images of the control group were directly analyzed and processed by professionals, while those of the observation group were processed by automatic segmentation technology. All the images were evaluated by the same team of senior imaging experts.  Figure 2 shows the definition of ISR.

### 2.3. The Improved Automatic Segmentation Algorithm

#### 2.3.1. Data Preprocessing

When the heart was scanned by CTA, many different tissues were involved, including the heart, bone, lung, and coronary artery [17, 18]. Different tissue densities were generated. The difference of Hounsfield unit (HU) values [19] was reflected in the CTA images. However, the CT values of coronary arteries that needed to be scanned were not markedly different from those of the surrounding tissues. To highlight the coronary arteries, it was necessary to preprocess the CTA images. In general, the CT values of coronary CTA ranged from 0 HU to 600 HU, and the window level and windowing were 300 HU and 600 HU, respectively. The relationship between them satisfied equations (1), (2), and (3):

(1) $$\begin{array}{c} \left\{\begin{array}{c} y=0\\ x\in \left(0,wl-\frac{ww}{2}\right) \end{array}\right), \end{array}$$

(2) $$\begin{array}{c} \left\{\begin{array}{c} y=128+\frac{256\cdot \left(x-wl\right)}{ww}\\ x\in \left[wl-\frac{ww}{2},wl+\frac{ww}{2}\right] \end{array}\right), \end{array}$$

(3) $$\begin{array}{c} \left\{\begin{array}{c} y=255\\ x\in \left(wl+\frac{ww}{2},600\right) \end{array}\right). \end{array}$$

In the above equations, *y* represents the HU value of CTA image output, *x* represents the HU value of CTA image input, *ww* represents the windowing of CTA image, and *wl* represents the window level of CTA image. Then, the CT values of coronary CTA images were reduced to 0–245 by data enhancement.

#### 2.3.2. Coronary CTA segmentation

The traditional region growth segmentation algorithm needed to manually set the initial point and threshold, so there was a great dependence. The region growth algorithm was combined with vascular similarity to improve the region growth and the accuracy of the segmentation algorithm. This algorithm includes three parts.

Firstly, the similarity features of blood vessels were extracted, which mainly involved the Hessian matrix [20] and the similarity function of blood vessels. The Hessian matrix of blood vessels was calculated by treating blood vessels as tubular structures. Then, three-dimensional data of vascular Hessian matrix were expressed as (7).

(4) $$\begin{array}{c} H_{\left(X-X\right)}=\left[I_{XX}\left(X\right),I_{XY}\left(X\right),I_{XZ}\left(X\right)\right], \end{array}$$

(5) $$\begin{array}{c} H_{\left(X-Y\right)}=\left[I_{YX}\left(X\right),I_{YY}\left(X\right),I_{YZ}\left(X\right)\right], \end{array}$$

(6) $$\begin{array}{c} H_{\left(X-Z\right)}=\left[I_{ZX}\left(X\right),I_{ZY}\left(X\right),I_{ZZ}\left(X\right)\right], \end{array}$$

(7) $$\begin{array}{c} H_{\left(X\right)}=\left[\begin{array}{c} H_{\left(X-X\right)}\\ H_{\left(X-Y\right)}\\ H_{\left(X-Z\right)} \end{array}\right]. \end{array}$$

In equations (4), (5), (6), and (7), a series of *I*_*xx*_*(X)* represented the second derivative of point *X* along the *X*, *Y*, and *Z* directions of the graph. To improve the determination of vascular scale, the algorithm also introduced multiscale filtering, namely, the convolution of original data and the Gaussian kernels of different variances. The Gaussian kernel was expressed as follows:

(8) $$\begin{array}{c} G_{\left(X,\alpha \right)}=\left(\frac{1}{{\left(\sqrt{2\pi \alpha^{2}}\right)}^{3}}\right)\cdot e^{-\left(\frac{{\left\|X\right\|}^{2}}{2\alpha^{2}}\right)}. \end{array}$$

In (8), *α* represents the variance, and *G* (*X*, *α*) represents that when the original data are at *X*, the variance is the Gaussian kernel of *α*. The Hessian matrix of the data of different scales was obtained by extracting the vascular features of different scales in the image through convolution. Then, the eigenvalue *β*_*q*_ (*q* = 1, 2, 3) was calculated, and the corresponding eigenvector was *χ*_*q*_(*q*=1,2,3). When *β*_*1*_>*β*_*2*_>*β*_*3*_, based on voxels in blood vessels, *β*_*3*_ would approach 0 infinitely, and *χ*_3_ represented the radial direction of the vessel. *β*_*1*_ and *β*_*2*_ would be close and equal infinitely, *χ*_1_ represents the tangential direction of the blood vessel, and *χ*_2_ represents the normal direction of blood vessels. The features of tubular structures were screened according to the eigenvalues. In accordance with the abovementioned calculation, some experts proposed the vascular similarity function under the eigenvalue, eigenvalue features, and vascular geometry features. The specific expression was as follows:

(9) $$\begin{array}{c} U_{r}\left(t\right)=\left\{\begin{array}{cc} 0, & \text{if }\beta_{1}>\frac{0}{\beta_{3}}>0,\\ \left(1-U_{1}\right)•U_{2}•\left(1-U_{3}\right), & \text{other} \end{array}\right). \end{array}$$

It was also expressed as (13).

(10) $$\begin{array}{c} S={\left\|H\right\|}_{F}=\sqrt{\sum_{i=1}^{3}\beta_{i}^{2}}. \end{array}$$

(11) $$\begin{array}{c} U_{1}=\exp-\left[\frac{{\left(\left|\beta_{2}\right|/\left|\beta_{3}\right|\right)}^{2}}{\left(2\varepsilon^{2}\right)}\right]. \end{array}$$

(12) $$\begin{array}{c} U_{2}=\exp-\left[\frac{{\left(\left|\beta_{1}\right|/\sqrt{\left|\beta_{2}\beta_{3}\right|}\right)}^{2}}{\left(2\phi^{2}\right)}\right]. \end{array}$$

(13) $$\begin{array}{c} U_{3}=\exp-\left[\frac{\left(S^{2}\right)}{\left(2\varphi^{2}\right)}\right]. \end{array}$$

*S* represents the Gaussian Blur in (8). *ε* and *ϕ* represent the threshold that controlled the linear filter. *φ* needed to determine the threshold according to the gray level of the image.

Secondly, the seed point was located, and the root node of the coronary artery was automatically located according to the significance of the ascending aorta and the connection with the coronary artery to achieve the automatic segmentation of the coronary artery. Due to the irregularity of the ascending aorta circle, the segmentation method under convolutional neural network (CNN) was adopted. The idea of CNN is encoding (convolution-feature extraction)-decoding (deconvolution-feature mapping) mode. In the training process of ascending the aorta section by this mode, the loss function was DiceLoss. It was expressed as

(14) $$\begin{array}{c} \text{DiceLoss}=1-\left[\left(2\sum_{j\in C}\left({\text{lab}}_{j}\cdot {\text{pre}}_{j}\right)+\frac{\text{smooth}}{\sum_{j\in C}{\text{pre}}_{j}}+\sum_{j\in C}{\text{lab}}_{j}+\text{smooth}\right)\right]. \end{array}$$

In (14), *C* represents a collection of pixels for the entire, *lab* represents the pixel label, and *pre* represents the predicted value of pixels. *Smooth* represents the constant in case that the denominator was zero.

The final part was the region growth. The conditions for the automatic implementation of region growth were provided by the abovementioned calculation. The specific steps of the region growth were as follows.

The first step was establishing the initial seed point.

The second step was fixing the voxel in the adjacent region of the seed point as the center and setting it as the point to be measured. It was calculated whether the growth conditions were satisfied. Then, the ones that were not satisfied were written down which were not calculated in the next growth. The other points that satisfied the requirements were cached.

The third step was extracting out one of the tested voxel points from the cache to update the initial seed points in the second step and repeat it.

The last step was to stop growing when the pixels to be measured satisfied the growth conditions when finished updating.

#### 2.3.3. Methods of Evaluation

Image enhancement, extraction of similarity features of vessels at different scales, segmentation based on CNN, and the segmentation effect of the overall segmentation algorithm were analyzed. Based on the segmentation accuracy of CNN, the error between the pixels at the corresponding position on the output image and the original label image was evaluated. The calculation method was shown in (15). In (16), the segmentation effect of the overall segmentation algorithm was measured by the average voxel error [21].

(15) $$\begin{array}{c} \text{Acc}=\left(\frac{1}{P}\right)\cdot \sum_{j\in C}\left(\frac{V_{i}}{G_{i}}\right). \end{array}$$

In (15), *P* represents the number of samples in the test set, *C* represents the collection of test set pixels, *V* represents the correct number of pixels in the predicted image, and *G* represents the number of pixels of positive samples in the annotation image.

(16) $$\begin{array}{c} \text{Error}=\left(\frac{1}{P}\right)\cdot \sum_{j\in C}\left(o_{i}-O_{i}\right). \end{array}$$

In (16), *P* represented the population prime point, *C* represented the whole data, *o* represented the voxel points to be compared, and *O* represented the standard voxel point.

### 2.4. Observation Indexes

- Two or more cardiovascular imaging physicians evaluated the CTA image quality of the two groups.  Table 1 shows the scoring criteria.
- The diagnostic sensitivity, specificity, positive predictive value, negative predictive value, and accuracy of CTA images of the two groups were evaluated based on the diagnostic results of CAG for coronary artery disease stenosis in postoperative review as the criteria.

### 2.5. Statistical Methods

SPSS 22.0 was employed for data statistics and analysis. The data were expressed as $\bar{x}$ ±*s*, and the two independent sample *t*-test was adopted for intergroup comparison. Percentage (%) or cases was how count data were expressed, and the intergroup comparison was tested by *χ*^2^. The difference was statistically considerable with *P* < 0.05.

## 3. Results

### 3.1. The Algorithm Performance

#### 3.1.1. The Effect of Image Enhancement

After enhanced processing, the CT value method of the coronary CTA image was compressed to 0–245 HU.  Figure 3 shows the effect of processing. The comparison between the coronary artery and the surrounding tissue was evidently enhanced. The coronary artery area was more prominent, while the surrounding tissue was observably reduced, which was more helpful to observe the lesion.

#### 3.1.2. Extraction of Similarity Features of Vessels of Different Scales

Figure 4 shows the fuzzy results of the Gaussian kernel with different variances (*α* = 0.5, 1, 2). With the increase of *α* value, the response of small structural features was weakened gradually. After several tests, the resulting images of *α* = 0.5, 1, and 2 were fused. The results showed that the details of various vessels in the fused images were reflected (Figure 4(e)).

#### 3.1.3. CNN Algorithm Segmentation Effect

The CNN algorithm was used to segment ascending aorta slices.  Figure 5 shows the segmentation effects of ascending aorta sections at different levels (if the highest layer was the first layer, Figure 5 was the first and second layer from top to bottom). After calculation, the segmentation accuracy of the CNN algorithm was 87.89%, which was at a high level.

#### 3.1.4. The Improved Growth Automatic Segmentation Effect

The improved automatic growth segmentation and traditional region growth segmentation were compared regarding the average voxel error (HU/voxel). The results showed that the average voxel error of the improved segmentation method was 1.8921 (HU/voxel), while that of the traditional region growth method was 7.10091 (HU/voxel). The average voxel error of the improved segmentation method was obviously lower than that of the traditional growth algorithm (*P* < 0.05) (Figure 6).

### 3.2. Comparison of Basic Data

Figure 7 shows the comparison of the basic data between the two groups. In the control group, 72.31% were males, and 27.69% were females. In the observation group, 66.15% were males, and 33.85% were females. The mean age of the control group was 61.34 ± 8.85 years old, and that of the observation group was 60.01 ± 9.65 years old. The mean diameter of the stents in the control group was 2.56 ± 0.21 mm, and that of the observation group was 2.96 ± 0.13 mm, without any significant difference (*p* > 0.05). It suggested that the study had certain feasibility.

### 3.3. The Score of Image Quality

The score results of the CTA image quality were as follows: the mean CTA score of the control group was (2.01 ± 0.73) and that of the observation group was (2.89 ± 0.11), which was notably higher than that of the control group (*p* < 0.05) (Figure 8). Figure 8(a) shows the CTA image of reexamination results 2 months after surgery of a 56-year-old male patient in observation group, and Figure 8(b) shows the CTA image of reexamination results two months and one week after surgery of a 60-year-old male patient in control group. According to Figure 8, the lumen and wall plaques of the coronary arteries in the observation group were more obvious than those in the control group (the lesions were inside the yellow circle).

### 3.4. Comparison of Diagnostic Efficacy of Restenosis

Figure 9 shows the restenosis diagnostic efficacy results of the two groups' CTA images. In the control group, CTA diagnostic sensitivity was 74.29% (26/35), specificity was 60% (18/30), positive predictive value was 68.42% (26/38), negative predictive value was 66.67% (18/27), and accuracy was 67.69% (44/65). In the observation group, CTA diagnostic sensitivity was 91.43% (32/35), specificity was 86.76% (26/30), positive predictive value was 88.89% (32/36), negative predictive value was 89.66% (26/29), and accuracy was 89.23% (58/65). Consequently, the restenosis diagnosis sensitivity, specificity, positive predictive value, negative predictive value, and accuracy of CTA images in the observation group were higher than those in the control group (*p* < 0.05).

## 4. Discussion

Region growth-based CTA images were used to diagnose restenosis after coronary stenting. To further improve the accuracy of image segmentation, the CNN algorithm and vascular similarity feature were combined to improve the region growth. The results showed that the segmentation accuracy of CNN algorithm could reach 87.89%, which was at a high level, indicating that the CNN algorithm had a good effect on image segmentation. Meijs et al. (2020) [22] proposed that the CNN algorithm had high performance in image segmentation. Moreover, the CNN segmentation algorithm was applied by many experts for CTA image diagnosis research, and the performance was affirmed [23–25]. However, in the extraction of vascular similarity features, the detailed vascular features could not be displayed with the gradual increase of the Gaussian kernel *α*. Nonetheless, after the fusion of the results of different scales, vessels of different sizes were revealed. Hence, multiscale vascular similarity feature extraction was more effective than single-scale vascular information extraction. The extraction of vascular similarity features involved the vascular similarity function, which was first proposed in 1998 and was widely used in the field of vascular segmentation [26]. Nevertheless, most of them were used for vascular segmentation of retinal images with high segmentation accuracy [27, 28]. Then, the improved region growth segmentation algorithm was compared with the traditional region segmentation algorithm. The results showed that the mean voxel error of the improved algorithm was manifestly lower than that of the traditional algorithm (1.8921 HU/voxel vs. 7.10091 HU/voxel) (*p* < 0.05). The smaller the mean voxel error was, the more accurate the segmentation result was. Consequently, the results indicated that the improved regional growth method could extract coronary arteries better. Region growth was a relatively common segmentation algorithm, which was involved in both magnetic resonance imaging (MRI) images [29] and CT images [30]. It was a segmentation method with great potential. The adoption effect of the improved method in clinical practice was explored.

Firstly, the quality scores of the two groups of CTA images were compared. The results showed that the mean score of CTA image in the observation group was higher than that in the control group (2.89 ± 0.11 points vs. 2.01 ± 0.73 points) (*p* < 0.05). Then, the diagnostic efficacy of CTA images in restenosis after coronary stenting was compared between the two groups. The results showed that the diagnostic sensitivity (91.43%), specificity (86.76%), positive predictive value (88.89%), negative predictive value (89.66%), and accuracy (89.23%) of the observation group were higher than those of the control group (*p* < 0.05). These results indicated that CTA images processed by an automatic segmentation algorithm were helpful to diagnose the restenosis after coronary stenting, and they also had good clinical adoption values, which reflected the adoption advantage of artificial intelligence (AI) in the field of medical imaging. In recent years, much attention has been paid to the adoption of segmentation algorithms in image processing, and lots of studies have shown that segmentation images are more conducive to the diagnosis of diseases. For instance, Liu et al. (2020) proposed that segmented MRI images could help doctors better observe a patient's heart health [31]. Furthermore, Pang et al. (2021) found that segmentation had great potential for clinical diagnosis and treatment of spinal diseases [32]. To sum up, the automatic segmentation algorithm was helpful to improve the diagnostic efficacy of CTA images with a good clinical adoption value.

## 5. Conclusion

In conclusion, the segmentation effect of the coronary CTA image was more precise by combining the CNN algorithm with the region growth algorithm of the vascular similarity feature. Besides, CTA images based on improved region growth segmentation algorithms had better clinical adoption value in the diagnosis of restenosis after coronary stenting. However, the type of patients selected in this study is relatively single, that is, only patients with single-vessel lesions, so it is not comprehensive enough and further comprehensive investigation is needed. The results of this study showed that the adoption of intelligent algorithms in the field of medical imaging had great potential, which was worth expecting and investigating.

## Figures and Tables

**Figure 1:** The evaluation criteria for ISR of CAG.

**Figure 2:** The evaluation criteria for ISR of CTA.

**Figure 3:** The effect of CTA data enhancement processing. (a) The original image; (b) the enhanced image.

**Figure 4:** The images of extraction effect of vascular similarity features under different values of *α*. (a) Original image; (b) the image with *α* = 0.5; (c) the image with *α* = 1; (d) the image with *α* = 2; (e) the fused image.

**Figure 5:** The segmentation effect of CNN algorithm. (a) The original image; (b) the labelling image; (c) the final effect image.

**Figure 6:** The effect images of regional growth segmentation. The image segmentation effect of (a) the improved region growth segmentation and (b) the traditional region growth segmentation.

**Figure 7:** Comparison of basic data.

**Figure 8:** The score results of CTA image quality. ∗The comparison between the two groups was of statistical significance, *p* < 0.05.

**Figure 9:** Comparison of diagnostic efficacy of CTA restenosis. ∗The comparison between the two groups was of statistical significance, *p* < 0.05.

**Table 1:** Scoring criteria of CTA image.

Score (point)	ISR	Variant	Artifact
**0**	Invisible structure	——	——
**1**	Visible structure	Obvious	Obvious
**2**	Still clear structure	Mild	Mild
**3**	Clear structure	Not found	Not found

## Data Availability

The data used to support the findings of this study are available from the corresponding author upon request.
